# Identification of Diagnostic Gene Markers and Immune Infiltration in Systemic Lupus

This article has been retracted.

**DOI:** 10.1155/2022/3386999

**Published:** 2022-05-10

**Authors:** Hongtao Hu, Chengsong He

**Affiliations:** Department of Rheumatology and Immunology, Southwest Medical University, Sichuan Province 646000, China

## Abstract

**Background:**

Systemic lupus erythematosus (SLE) is an autoimmune disease involving multiple organs, with atypical clinical manifestations and indefinite diagnosis and treatment. So far, the etiology of the disease is not completely clear. Current studies have known the interaction of genetic system, endocrine system, infection, environment, and other factors. Due to abnormal immune function, the human body, with the participation of various immune cells such as T cells and B cells, abnormally recognizes autoantigens, so as to produce a variety of autoantibodies and combine them to form immune complexes. These complexes will stay in the skin, kidney, serosa cavity, large joints, and even the central nervous system, resulting in multisystem damage of the body. The disease is heterogeneous, and it can show different symptoms in different populations and different disease stages; patients with systemic lupus erythematosus need individualized diagnosis and treatment. Therefore, we aimed to search for SLE immune-related hub genes and determine appropriate diagnostic genes to provide help for the detection and treatment of the disease.

**Methods:**

Gene expression data of whole blood samples of SLE patients and healthy controls were downloaded from the GEO database. Firstly, we analyzed and identified the differentially expressed genes between SLE and the normal population. Meanwhile, the single-sample gene set enrichment analysis (ssGSEA) was used to identify the activation degree of immune-related pathways based on gene expression profile of different patients, and weighted gene coexpression network analysis (WGCNA) was used to search for coexpressed gene modules associated with immune cells. Then, key networks and corresponding genes were found in the protein-protein interaction (PPI) network. The above corresponding genes were hub genes. After that, this study used receiver operating characteristic (ROC) curve to evaluate hub gene in order to verify its ability to distinguish SLE from the healthy control group, and miRNA and transcription factor regulatory network analyses were performed for hub genes.

**Results:**

Through bioinformatics technology, compared with the healthy control group, 2996 common differentially expressed genes (DEGs) were found in SLE patients, of which 1639 genes were upregulated and 1357 genes were downregulated. These differential genes were analyzed by ssGSEA to obtain the enrichment fraction of immune-related pathways. Next, the samples were selected by WGCNA analysis, and a total of 18 functional modules closely related to the pathogenesis of SLE were obtained. Thirdly, the correlation between the above modules and the enrichment fraction of immune-related pathways was analyzed, and the turquoise module with the highest correlation was selected. The 290 differential genes of this module were analyzed by GO and KEGG. The results showed that these genes were mainly enriched in coronavirus disease (COVID-19), ribosome, and human T cell leukemia virus 1 infection pathway. The 290 DEGs with PPI network and 28 genes of key networks were selected. ROC curve showed that 28 hub genes are potential biomarkers of SLE.

**Conclusion:**

The 28 hub genes such as RPS7, RPL19, RPS17, and RPS19 may play key roles in the advancement of SLE. The results obtained in this study can provide a reference in a certain direction for the diagnosis and treatment of SLE in the future and can also be used as a new biomarker in clinical practice or drug research.

## 1. Introduction

Systemic lupus erythematosus is a common autoimmune disease that causes pathogenic autoantibodies and immune complexes to form and mediate organ and tissue damage. Clinically, there are often multiple system involvement manifestations, and the early symptoms are often atypical, such as fever, fatigue, facial erythema, hair loss, serositis, and joint pain. Proteinuria, edema, and even renal failure may occur when the renal system is involved, and endocarditis, arrhythmia, and myocardial infarction may occur in the cardiovascular system. Pulmonary interstitial lesions often occur in the lungs. The blood system may show decreased hemoglobin, leukocytes, and platelets during the active period of the disease. The etiology of the disease includes genetic factors, environmental factors, and the role of estrogen. The disease mainly affects women, especially women of childbearing age. The proportion of men and women is about 2 : 8 to 1 : 9. At present, the mainstream treatment methods include glucocorticoids and immunosuppressants. In recent years, biological agents such as belimumab have emerged, and the treatment effect is relatively better. However, it is difficult to diagnose the disease in the early stage, and many diagnostic criteria have low sensitivity. Most of the patients in the acute stage died of severe multiple organ damage and infection caused by SLE, and most of them died of chronic renal insufficiency and adverse drug reactions in the long term. Therefore, it is urgent to further develop the diagnostic markers and therapeutic targets of SLE, so as to provide new methods for the treatment and intervention of patients.

Relevant studies have shown that the two most significant characteristics of SLE are the breaking of immune balance and the abnormal production of autoantibodies. In the pathogenesis of SLE, in addition to the innate immune system, the more important is the participation of the acquired immune system [1]. There are two ways to activate the innate immune system: Toll-like receptor (TLR) dependent and TLR independent. If the cell dies, it will release its DNA and RNA outside the cell, thus starting a chain reaction, so that the membrane-bound TLR (TLR2, 4, 6) is activated, leading to the downstream interferon regulatory family (IRF-3), and NF-*κ*B and MAP kinase are activated and act as transcription factors to produce proinflammatory mediators such as IFN-b [2]. Antigen-presenting cells play their role in presenting the antigens of apoptotic and damaged cells to T cells. T cells activate autoreactive B cells through the production of CD40L and cytokines, resulting in the production of autoantibodies. It can cause disease through direct or indirect action. First, they directly bind to the autoantigens of target organs, and second, their induced immune complexes pass through Fc*γ*R that activates inflammatory mediators (cytokines) or complement system, resulting in changes in cell function [3]. At the same time, B cells also play the role of antigen presentation and activate T cells, thus forming a vicious cycle of mutual activation of B and T cells [4]. However, systemic lupus erythematosus (SLE), as a highly hereditary autoimmune disease in the world, has obvious heterogeneity. It has different prevalence, clinical manifestations, and prognosis in terms of gender, age, and population [5]. Different patients, even at different stages of the same patient, have different affected systems. It is necessary to weigh the risks and benefits of clinical treatment according to the tolerance of patients with different physique and then select an individualized medication scheme.

At present, the heterogeneity of SLE can be explained by analyzing the human immune profiling [6]. From the multidimensional analysis of immune cells and the identification of relevant immune subsets of the disease, or transcriptome analysis, we can find the characteristics of gene network, deeply understand the pathological mechanism and heterogeneity of the disease, and find new biomarkers. This can not only realize the precision medical treatment of SLE but also improve and guide the clinical diagnosis and treatment of SLE in the future [3]. Therefore, this study starts with the immune cell infiltration of SLE, looks for the immune-related genes of SLE, determines the appropriate diagnostic gene markers, and provides inspiration for the future detection and treatment of the disease.

## 2. Research Materials and Methods

### 2.1. Data Source

Gene expression profiles of whole blood samples from 292 SLE patients and 20 control individuals in GSE45291 were downloaded from the GEO database (GPL13158 platform, Affymetrix HT HG-U133+ PM Array).

### 2.2. Acquirement of Differentially Expressed Genes (DEGs)

Generally, all the microarray data after normalization were analyzed by R software.

R package “limma” was used to identify differentially expressed mRNAs between SLE and control samples with ∣log_2_FC | >1 and adj. *p* val < 0.05 as the threshold (PMID: 25605792).

### 2.3. Functional Annotation and Pathway Enrichment Analysis

To reveal the functions of DEGs, GO annotation (PMID: 27899567) and KEGG enrichment (PMID: 10592173) analyses were conducted using the “clusterProfiler” package. For each gene, its basic function is based on its protein domain and the research literature. We can roughly know what kind of function a gene has. GO and KEGG are databases of gene-related functions stored based on different classification ideas. GO annotation describes what our differential genes are mainly related to from three levels: biological process (BP), cellular component (CC), and molecular function (MF). In addition to the annotation of human gene pathways, we also know the database of human gene pathways. KEGG is a kind of a path-related database. Adj. *p* val < 0.05 was considered statistically significant.

### 2.4. Analysis of Immune Infiltration

ssGSEA can analyze the pathways enriched by gene expression in each sample, so as to analyze the activation degree of specific pathways; the gene sets are classified from the following three aspects: common biological function, chromosome localization, and physiological regulation. We used it to analyze immune cell-related pathways in SLE patients and healthy controls. ssGSEA, as its name suggests, is a special GSEA. It mainly proposes an implementation method for single-sample unable to do GSEA. In principle, it is similar to GSEA. The difference is that GSEA needs to prepare the expression profile file, GCT, calculate the rank value of each gene according to the expression profile file, and then conduct subsequent statistical analysis.

### 2.5. Weighted Gene Coexpression Network Analysis (WGCNA)

WGCNA R package was used to construct the coexpression network (PMID: 19114008). Firstly, the Euclidean distance of expression quantity is used to cluster the samples and check whether there are outliers in the samples. Then, the coexpression network is obtained by using the automatic network construction function. Then, pickSoftThreshold is used to calculate the best soft threshold for filtering *β*. According to the rules of the algorithm source literature (PMID: 19114008), select the appropriate value as the soft threshold to identify the coexpression module again, select the significantly different immune-related pathways, and analyze the correlation between each module and the enrichment fraction of immune-related pathways. Finally, the gene modules related to immune infiltrating cells were identified. Extract the corresponding module gene information for GO and KEGG analyses again.

### 2.6. Protein-Protein Interaction (PPI) Network Construction

We constructed the PPI network by the STRING database (PMID: 25352553). Then, a visualized PPI network was created by Cytoscape (PMID: 14597658). By using MCODE plugin, the key module and the genes in the key module were screened from the whole network.

### 2.7. Validation of Hub Genes

In order to verify the importance of hub gene to SLE and evaluate whether it has the ability to distinguish SLE patients from control group, we analyzed it by drawing ROC curve and calculated AUC using “proc” software package (PMID: 21414208).

### 2.8. Multifactor Regulation Network Construction

We used NetworkAnalyst (PMID: 30931480) and miRNet (PMID: 30421406) databases to predict the TFs and miRNAs of hub genes. Hub genes and their miRNAs and TFs were integrated into a regulatory network and visualized using the Cytoscape software.

## 3. Results

### 3.1. Identification of Differentially Expressed Genes (DEGs)

Differential analysis of the microarray results of gse45291 showed that 1357 downregulated genes and 1639 upregulated genes were detected, with a total of 2996 differentially expressed genes detected as shown in Figure 1(a).  Figure 1(b) shows the expression of the top 10 DEGs by a heat map.

### 3.2. GO Annotation and KEGG Pathway Enrichment Analysis of DEGs

To obtain a deeper insight into the biological roles of these 2996 DEGs, GO annotation and KEGG enrichment analyses were conducted using “clusterProfiler” package. GO-BP analysis showed that these 2996 DEGs were significantly enriched in neutrophil activation, neutrophil-mediated immunity, and neutrophil activation involved in immune response (Figure 2(a)). For GO-CC analysis, presynapsis, cell-substrate connection, and neuronal cell body are the three terms with the most enrichment (Figure 2(b)). Deoxyribonucleic acid-binding transcriptional activation activity, binding transcriptional activation activity of RNA polymerase II-specificity, and cyclin-dependent protein kinase activity are the top three terms in MF analysis (Figure 2(c)). In addition, the top three markedly enriched pathways for these 2996 DEGs were coronavirus disease (COVID-19), Epstein-Barr virus infection, and human T-cell leukemia virus 1 infection (Figure 2(d)). Combined with KEGG and GO results, it can be seen that most of DEGs are immune-related genes in the SLE patients and controls, which is consistent with the pathological characteristics of SLE.

### 3.3. Immune Infiltration Analyses

We first investigated the difference in immune infiltration between SLE and control in 28 immune cell-related pathways by ssGSEA.  Figure 3(a) summarizes the results obtained from 20 normal controls and 292 SLE patients. Compared with normal tissue, SLE tissue generally contained a higher proportion of type 2 T helper cell, natural killer cell, and immature dendritic cell, whereas the natural killer T cell, memory B cell, and effector memory CD8 T cell were relatively lower (Figure 3(b), *p* < 0.05) in SLE samples.

### 3.4. Weighted Coexpression Network Construction and Identification of Key Modules

This study used Pearson correlation coefficient to cluster the samples and check whether there are outliers in the samples. After removing one outlier, draw a sample clustering tree (Figures 4(a)–4(b)) and refer to the rules of the algorithm source literature (PMID: 19114008); we set the soft threshold to 5 to construct a scale-free network (Figure 4(c)). Then, eighteen modules were identified based on average hierarchical clustering and dynamic tree clipping (Figure 4(d)). The turquoise module was highly related to activated CD8+ T cell, immature B cell, type 2 T helper cell, immature dendritic cell, and effector memory CD8 T cell. Thus, this module was selected for further analysis (Figure 4(e)).

### 3.5. GO and KEGG Enrichment Analyses of Immune-Related Genes

We cross-linked turquoise module genes and DEGs to obtain 290 immune-related genes (Figure 5).

Next, the immune-related genes were enriched and analyzed by GO analysis and KEGG analysis. The results of these analyses showed that those genes were mainly enriched in the biological process of ribonucleoprotein complex biogenesis. As for the cellular component, the genes were mainly enriched in cell-substrate junction. Finally, regarding molecular function, the genes were mainly enriched in structural constituent of ribosome (Figures 6(a)–6(c)). KEGG analysis showed that these genes were significantly activated in the signal pathway involved in coronavirus disease (COVID-19), followed by ribosome and human T cell leukemia virus 1 infection (Figure 6(d)).

### 3.6. Construction of PPI Network

The PPI network of 290 immune-related genes was constructed using the STRING database and visualized by Cytoscape (Figure 7(a)). The key module was obtained using MCODE, and 28 genes in the key module were selected as hub genes (Figure 7(b)). The genes in red are upregulated in SLE patients compared with normal controls, and the genes in blue are downregulated.

### 3.7. Hub Gene Validation

The results indicated that all hub genes were significantly differentially expressed between the control and SLE groups (Figure 8(a)). Next, ROC curve was plotted and the area under the curve (AUC) was calculated. The AUC of 28 hub genes were all greater than 0.7 (Figure 8(b)), and RPS7 has the higher diagnostic value as a biomarker, whose area under curve reached 0.987.

### 3.8. Multifactor Regulation Network Construction

By using the miRNet and NetworkAnalyst databases, the miRNAs-hub genes (Figure 9(a)) and TFs-hub genes (Figure 9(b)) networks were constructed by the Cytoscape software. In order to facilitate the selection of important miRNAs, miRNAs targeting at least 4 hub genes were selected for the network. Finally, the network includes 26 hub genes, 42 miRNAs, and 51 TFs.

## 4. Discussion

In order to find new biomarkers as diagnostic markers or therapeutic targets for SLE, so as to carry out individualized and differentiated precision medicine for the disease, in this study, bioinformatics analysis was used to download the gene expression detection data of whole blood samples from SLE patients and healthy controls from the GEO database, and limma package was used to identify the differentially expressed genes between SLE and normal population.

We enriched 2996 differentially expressed genes by GO and KEGG, which showed that the differentially expressed genes were mainly enriched in infection and immune-related pathways. On the other hand, ssGSEA analyzed the different immune cell-related pathways between SLE patients and healthy controls, screened key modules through WGCNA, obtained 290 immune-related differential genes, and enriched 290 genes with GO and KEGG again. GO analysis showed that it was mainly enriched in immunity, cell membrane structure, and gene transcription regulation pathway. KEGG analysis showed that these genes were significantly activated in the signal pathways involved in coronavirus (COVID-19), ribosome, and human T cell leukemia virus 1 infection. Among them, 27 genes are involved in ribosome and COVID-19 pathway.

Currently, humans are fighting against novel coronavirus pneumonia caused by SARS-CoV-2 new coronavirus. Susceptible populations include people with immunodeficiency due to potential diseases. As a key factor, immune response is involved in the disease progression, severity, and clinical outcome of COVID-19, as well as the human body's defense against the virus [7]. Because SLE is a common autoimmune disease, it seems that SLE patients are more vulnerable to COVID-19, which may be patients with autoimmune diseases (such as lupus) have abnormal immune response and the immune tolerance mechanism is broken. In addition, the current mainstream treatment scheme is to inhibit immune function through drugs, such as hormones and immunosuppressants. The joint participation of these factors will lead to the further increase of immune deficiency status and infection risk [7]. However, it is still unknown how SLE patients will respond to COVID-19 infection and whether these patients will increase the risk of infection, and the current data show that few COVID-19 patients are complicated with SLE [8]. Previous studies have shown that a particularly important link in the pathogenesis of SLE is the abnormal participation of T cells and B cells due to normal immune dysfunction. SLE is mainly mediated by abnormal B cells and their plasma cells. One of the characteristics of SLE is that B cells produce too many autoantibodies, resulting in systemic inflammation. However, the fact is that abnormal T cells are identically essential key promoters of systemic inflammation observed, because they will participate in the process of stimulating the proliferation, maturation, and differentiation of B cells, so as to enhance the production and conversion of autoantibodies in SLE. Relevant studies have confirmed that in this autoimmune disease, the overactivation of T cells is related to COVID-19, because stimulating the adaptive immune system after infection may have more serious consequences for SLE patients [9].

Interestingly, relevant studies show that the two diseases show significant differences in specific population distribution and different genders. Men were hospitalized and died more because of COVID-19, while female SLE had a higher incidence rate. That is, men tend to be infected, while women are more vulnerable to autoimmune diseases [10]. The proposed explanation for this difference is that first, it comes from heredity, X chromosome inactivation, also known as lyonization, refers to the phenomenon that female mammals will not produce twice the gene product because they have two X chromosomes, and one of the two X chromosomes in the cell will lose activity. In the process, the X chromosome will be packaged into heterochromatin, and then, the gene function will be inhibited and silenced. Therefore, they can express only one gene on the X chromosome like males. Existing studies have confirmed that there are immune-related genes on the X chromosome.

However, some genes may not be silenced, resulting in noninactivation, and eventually produce gene products expressed by double alleles [10]. The increased activation of T cells and B cells in women has been confirmed to be related to the biallelic expression of immune-related genes, which shows that women are more likely to suffer from SLE from another perspective and shows the difference between men and women in COVID-19 immune response. The second explanation for the observed gender bias is derived from the role of sex hormones: estrogen produces immune activation, while androgens such as testosterone produce immunosuppression [11]. The microbiota will be affected by estrogen and increase diversity, leading to the upregulation of some cytokines [10]. On the contrary, male testosterone significantly reduces the aggressiveness of human immune response by upregulating IL-10 and inhibiting the expression of inflammatory factors such as TNF, IL-6, and IL-1 through activated macrophages [10]. Specifically, sex hormones may increase the probability of inflammation in women, and the ability of hormone factors to improve the clearance of infection may also increase the possibility of autoimmune diseases in women [10], and the stronger immune response may be additionally involved by genetic components and diverse microbiota, which leads to more proinflammatory cytokines in women than in men [10]. It has been confirmed that the activation of CD4 T cells and the expression of proinflammatory cytokines IL-1B and IFN-g are related to the level of estrogen in women. Intensified expression of proinflammatory cytokines in women may encourage the antivirus activity against coronavirus, although it promotes the immune imbalance in autoimmune diseases.

However, lupus and COVID-19 also have many similarities in clinical manifestations and pathological mechanisms. Both of them are manifested in multiple organ complications such as interstitial pneumonia, myocarditis, joint pain, hemocytopenia, and hemophagocytic lymphohistiocytosis [12]. At present, in patients infected with coronavirus, immunosuppressants have been used as one of the possible means to inhibit inflammation and reduce respiratory distress in patients with acute respiratory distress syndrome (ARDS) due to many disease characteristics of SLE and COVID-19 [13]. Therefore, the treatment idea of SLE can inspire the current treatment of COVID-19 to a certain extent, indicating that we can start from the direction of immunosuppression. This study uses bioinformatics technology; finding the genes involved in COVID-19 pathway in SLE patients may further explore more links between lupus and COVID-19.

In order to further find the key genes affecting SLE, we screened the core module through PPI, and ROC identified biomarkers that can be used to diagnose SLE. Finally, the TF and miRNA networks related to hub gene were constructed. ROC recognition results show that the gene RPS7 (ribosomal protein S7) has the best discrimination performance, and its area under ROC curve reaches 0.987. The gene is a component of the 40s subunit, which encodes a ribosomal protein. The protein belongs to the s7e family of ribosomal proteins and is located in the cytoplasm. Therefore, RPS7 is a protein coding gene. At present, it is known that the related diseases involved in RPS7 include Diamond Black fan anemia 8 and Diamond Black fan anemia. GO annotations related to this gene are RNA binding and structural components of ribosomes, respectively. Related pathways involved include HIV life cycle and viral mRNA translation. The hub gene miRNA regulatory network (RPL11, RPS4x, and RPL39) and hub gene transcription factor regulatory network (RPL11, RPS4x, and RPL39) were upregulated in SLE patients compared with normal controls.

Relevant literature shows that in the pathogenesis of systemic vasculitis, ribosome-related genes enriched in ribosomal pathway, such as RPL31, RPS3a, and RPL9, interact with each other which lead to the occurrence of the disease [14]. It is also reported that when the cell potassium content decreases, it can inhibit the ribosome function, resulting in the processing of interleukin- (IL-) 1B and inflammatory activation [14]. Through this discovery, we can speculate that ribosomal protein-related genes involved in the upregulation of ribosomal pathway may promote inflammation by regulating cellular potassium. We have detected a decrease in blood potassium in patients with Kawasaki disease or nodular polyarteritis [15, 16]. Unfortunately, there is no relevant evidence to show the relationship between these genes and SLE, and this study shows that these genes are downregulated in SLE patients. However, interestingly, these genes are also enriched in the intestinal immune network produced by IgA and the pathway of systemic lupus erythematosus, and their role in SLE needs to be further studied.

Another study on neuropsychiatric lupus erythematosus (hereinafter referred to as NPSLE) and SLE showed that the positive rates of RPLP0, RPLP1, RPLP2, and SS-A autoantibodies in the NPSLE group were significantly higher than those in the non-NPSLE group or control group. One theory is that there is a strong correlation between the autoantibody titer of cerebrospinal fluid and serum samples, which suggests that the autoantibody found in cerebrospinal fluid may be caused by the leakage of damaged blood-brain barrier in the blood [17]. However, this study suggests that related genes are downregulated in SLE patients. The possible reasons are as follows: (1) It has been reported that anti-RPLP0, anti-RPLP1, and anti-RPLR2 autoantibodies have been found in a large number of cerebrospinal fluid samples of SLE patients [18, 19]. (2) The data source of this study is the whole blood gene expression test data of SLE patients, not the cerebrospinal fluid of patients, considering that NPSLE includes more autoantibodies, which leads to the occurrence of the disease. (3) The literature also points out that the prevalence of disease-related autoantibodies in cerebrospinal fluid of SLE patients is low, and the prevalence of disease-related autoantibodies in the NPSLE group and the non-NPSLE group is <45%. Only a few autoantibodies were positive, the positive rate was between 30% and 45%, and the positive rate of most antibodies was between 15% and 30%. This result is consistent with most autoantibody studies reported in the past on SLE. Therefore, more multiple detection and clinical experiments of autoantibodies are needed to prove the correlation between RPLP0, RPLP1, and RPLP2 and NPSLE and SLE [17].

There are other reports pointed out that RPLP0 (acid ribosomal protein P0) was used as the target antigen identified from 35 kD protein. Lupus-like histological changes occurred after intradermal injection induced by purified serum anti-RPLP0 antibody. The experiment further showed that the level of anti-RPLP0 antibody in SLE patients was significantly higher than that in the healthy control group and decreased with skin recovery. In addition, the antibody level was positively correlated with leukopenia and C3 deficiency. To some extent, the active phase of arthritis and SLE is also related to the increase of anti-RPLP0 antibody level [20]. The results show that the immune response mediated by serum anti-RPLP0 antibody plays a key role in the pathogenesis of SLE. This is consistent with the results of our study.

The three upregulated genes of hub gene (rps7, rpl39, and rpl1) in this study suggest that they may be closely related to the pathogenesis of SLE, but the relationship between hub gene and SLE has not been studied. And the three upregulated genes involved in the pathway include viral mRNA translation, rRNA processing in nuclei and cells, transcription and replication of influenza virus RNA, and the life cycle of HIV. It is necessary to further study their role in the development of SLE.

This study has some limitations. Firstly, the selected sample size is relatively small, and more sample size is needed for future research. Secondly, limited by time and funds, this study only uses bioinformatics methods. As a supplement to this study, the expression changes of DEGs at mRNA level or protein level can be detected by RT-PCR or Western blot and even supplemented with clinical samples or animal level experiments. We can also knock down/overexpress the screened genes, carry out functional experiments, and verify the results with the functional enrichment of biological information technology.

## 5. Conclusion

In conclusion, this study identified 28 characteristic genes of immune cell-related pathways and identified many key genes related to SLE. In addition, it plays an significant role in the occurrence, development, and prognosis of SLE. These results provide new inspiration in the direction of molecular basis for us to better understand the pathogenesis of SLE and provide valuable new biomarkers for the diagnosis and treatment of SLE. In the future, we can explore new diagnostic methods and therapeutic drugs of SLE from a relevant perspective.

## Figures and Tables

**Figure 1:** (a) Volcano plot for the differential expression analysis. (b) Heat map for DEGs.

**Figure 2:** (a) GO enrichment of DEGs for biological process. (b) GO enrichment of DEGs for cellular component. (c) GO enrichment of DEGs for molecular function. (d) KEGG enrichment of DEGs.

**Figure 3:** (a) Heat map for the enrichment score of immune-related pathways. (b) Box diagram for the enrichment score of immune-related pathways.

**Figure 4:** (a, b) Sample clustering and detecting outliers. (c) Soft threshold selection. (d) WGCNA modules. (e) Correlation between coexpression modules and immune-related pathways.

**Figure 5:** Intersection between genes in module turquoise and DEGs.

**Figure 6:** (a–c) GO enrichment of the 290 genes for biological process, cellular component, and molecular function. (d) KEGG enrichment of the 290 genes.

**Figure 7:** (a) PPI network of 290 DEGs in module turquoise. (b) PPI subnetwork of hub genes.

**Figure 8:** (a) Expression of hub genes. (b) ROC of hub genes on determining SLE patients from the normal control.

**Figure 9:** (a) miRNA regulation network of hub genes. (b) Transcription factor regulation network of hub genes.

## Data Availability

No data were used to support this study.
